The article "Construction and Evaluation of Prognosis Prediction Model for Patients with Brain Contusion and Laceration Based on Machine Learning" was published in 2022. Journal: Comput Math Methods Med.

# Construction and Evaluation of Prognosis Prediction Model for Patients with Brain Contusion and Laceration Based on Machine Learning

**DOI:** 10.1155/2022/4311434

**Published:** 2022-05-12

**Authors:** Shaoquan Li, Limei Bai, Zhixia Zheng

**Affiliations:** Department of Neurosurgery, Cangzhou Central Hospital, Hebei 061000, China

## Abstract

**Objective:**

Finding valuable risk factors for the prognosis of brain contusion and laceration can help patients understand the condition and improve the prognosis. This study is aimed at analyzing the risk factors of poor prognosis in patients with brain contusion after the operation.

**Methods:**

A total of 136 patients with cerebral contusion and laceration combined with cerebral hernia treated by neurosurgical craniotomy in our hospital were retrospectively selected and divided into a training set (*n* = 95) and a test set (*n* = 41) by the 10-fold crossover method. Logistic regression and back-propagation neural network prediction models were established to predict poor prognosis factors. The receiver operating characteristic curve (ROC) and the calibration curve were used to verify the differentiation and consistency of the prediction model.

**Results:**

Based on logistic regression and back-propagation neural network prediction models, GCS score ≤ 8 on admission, blood loss ≥ 30 ml, mannitol ≥ 2 weeks, anticoagulants before admission, and surgical treatment are the risk factors that affect the poor prognosis of patients with a cerebral contusion after the operation. The area under the ROC was 0.816 (95% *CI* 0.705~0.926) and 0.819 (95% *CI* 0.708~0.931), respectively.

**Conclusion:**

The prediction model based on the risk factors that affect the poor prognosis of patients with brain contusion and laceration has good discrimination and accuracy.

## 1. Introduction

In recent years, brain contusion and laceration have been increasing with the continuous renewal of transportation [1]. In traffic accidents, the head and neck are some of the most seriously injured parts. Severe traumatic brain injury (TBI) can lead to brain contusion and laceration, mainly manifested by the cooccurrence of contusion and laceration tissues and intracranial edema, with high mortality and disability rates [2]. Brain contusion and laceration refer to two diseases: brain contusion and brain laceration. If the patient only suffers from brain parenchyma injury and the pia mater is not damaged, it is brain contusion. In addition to brain parenchyma damage, it is brain laceration if the patient's pia mater is torn. Brain contusion and laceration refer to the phenomenon that both brain contusion and brain laceration coexist in the patient [3].

The article "Construction and Evaluation of Prognosis Prediction Model for Patients with Brain Contusion and Laceration Based on Machine Learning" was published in 2022. Journal: Comput Math Methods Med.

Cerebral contusion and laceration mean that patients are prone to increase intracranial pressure and have a greater chance of forming cerebral hernias [4]. Existing research generally advocates that surgical treatment should be recommended on the premise that patients have surgical indications. A craniotomy is an effective treatment, but it is difficult to handle and has a high mortality rate [5]. Brain contusion and laceration in primary TBI are one of the most common diseases. The influencing factors of prognosis of patients with severe traumatic brain injury are issues that scholars pay extensive attention [6]. Progressive brain contusion and laceration are related to many factors. Through early analysis of the relevant factors, we can obtain the valuable risk factors for the prognosis, which is of great significance to helping patients with brain contusion and laceration to study the condition and improve the prognosis [7, 8]. Therefore, it is helpful to improve the prognosis of patients with brain contusion by identifying the risk factors that affect the poor prognosis after the operation and giving appropriate treatment at an early stage.

Machine learning algorithm has unique advantages in dealing with high-dimensional variables, complex interactions, and nonlinear relationships among variables [9–12]. The prediction analysis of machine learning has been widely used in the biomedical field [13–15]. Based on logistic regression and neural network, this paper constructs a prediction model to study the high-risk factors of poor prognosis in brain contusion and laceration patients. The results can provide suggestions for the surgical plan and postoperative prognosis.

## 2. Methods

### 2.1. General Data

A total of 136 patients with brain contusion and laceration admitted to our hospital from 2016 to 2021 were selected as the research object. There were 102 males and 34 females, aged from 18 to 65 (57.54 ± 11.43) years. All patients meet the clinical diagnostic criteria of brain contusion and laceration, and all patients have signed the research consent before participating in this study. Inclusion criteria are as follows: (1) there is a clear history of traumatic brain injury, and a head CT examination is performed to confirm the diagnosis. (2) There are indications for craniotomy. Exclusion criteria are as follows: (1) severe dysfunction of other organs, (2) suffering from blood system diseases, (3) patients complicated with a malignant tumor, and (4) suffering from mental illness.

### 2.2. Collection of Predictive Variables

The gender, age, Glasgow coma scale (GCS) score, blood loss, the application time of mannitol, whether anticoagulants were used before admission, and operation methods were collected.

The article "Construction and Evaluation of Prognosis Prediction Model for Patients with Brain Contusion and Laceration Based on Machine Learning" was published in 2022. Journal: Comput Math Methods Med.

### 2.3. Construction of Machine Learning Model

Logistic regression is the most commonly used statistical model for predicting the outcome variable as a binary variable, which is often used in data mining, automatic diagnosis of diseases, and other fields. One result of the dichotomous response variable *Y* is denoted as “success,” denoted by 1. The other result is denoted as “failure,” denoted by 0 [16]. Its general form is as follows:

(1) $$\begin{array}{c} \text{Log}it\left(P\right)=\log\left(\frac{P}{1-P}\right)=a+b_{1}x_{1}+b_{2}x_{2}+\cdots +b_{m}x_{m}. \end{array}$$

*x*_1_, *x*_2_,…, *x*_*m*_ are predictors, and *b*_1_, *b*,…, *b*_*m*_ are regression coefficients of *m* predictors.

The probability *p* of the predicted event can be obtained by simple transformation of formula (1).

(2) $$\begin{array}{c} P=\frac{\exp\;\left(a+b_{1}x_{1}+b_{2}x_{2}+\cdots +b_{m}x_{m}\right)}{1+\exp\;\left(a+b_{1}x_{1}+b_{2}x_{2}+\cdots +b_{m}x_{m}\right)}. \end{array}$$

### 2.4. Artificial Neural Network

The neural network model used in this paper is the back-propagation neural network (BPNN). It has a good ability to solve nonlinear problems, and it is the most popular and classic neural network model so far [17]. As a supervised learning process, BPNN algorithm repeatedly replaces the weights and thresholds of network connection with known input and output sample data so that the network's output is closer to the expected output [18]. As far as the whole neural network is concerned, a learning process is completed by two subprocesses of forwarding propagation of input data and backward propagation of error [19]. The classical BPNN structure is shown in Figure 1.

There are *n* neurons in the input layer, *p* neurons in the hidden layer, and *q* neurons in the output layer. Define the input vector as follows:

(3) $$\begin{array}{c} X=\left(x_{1},x_{2},\cdots ,x_{n}\right). \end{array}$$

Selecting randomly the *k*-th input sample and its corresponding expected output:

(4) $$\begin{array}{c} x\left(K\right)=\left(x_{1}\left(k\right),x_{2}\left(k\right),\cdots ,x_{n}\left(k\right)\right). \end{array}$$

Calculating the input and output of neurons in the hidden layer:

(5) $$\begin{array}{c} {hi}_{h}\left(k\right)=\overset{n}{\underset{i=1}{\sum }}w_{ih}x_{j}\left(k\right)-b_{h}h=1,2,\cdots ,p. \end{array}$$

Finally, calculating the global error:

(6) $$\begin{array}{c} E=\frac{1}{2m}\overset{m}{\underset{k=1}{\sum }}\overset{q}{\underset{o=1}{\sum }}{\left(d_{o}\left(k\right)-y_{o}\;\left(k\right)\right)}^{2}. \end{array}$$

All patients were divided into a training set (*n* = 95) and a test set (*n* = 41) by stratified random sampling. The ratio of the training set to the test set is about 7 : 3. The 10-fold crossover method is used to validate the data. The advantage of this method is that all data are used in the training set and the test set, and each data set is divided into independent verification. The specific process is shown in Figure 2.

The article "Construction and Evaluation of Prognosis Prediction Model for Patients with Brain Contusion and Laceration Based on Machine Learning" was published in 2022. Journal: Comput Math Methods Med.

### 2.5. Statistical Analysis

The measurement data is expressed by $\bar{x\pm s}$, the data accords with normal distribution, the comparison between groups adopts an independent sample *t*-test, and the counting data is expressed by percentage. The *Chi-*square test was used to analyze the differences between different groups, and *P* < 0.05 means the difference is statistically significant.

## 3. Results

### 3.1. Comparison of Predictive Variables Influencing the Prognosis between Two Sets

There was no significant difference between the training set and test in gender, age, admission GCS score, blood loss, the application time of mannitol, use of anticoagulants within 1 week before admission, treatment methods, midline shift distance and brain contusion, and laceration volume (*P* > 0.05), as shown in Figure 3.

### 3.2. Logistic Regression Analysis of Predictive Variables of Postoperative Prognosis

Logistic regression analysis showed that GCS score ≤ 8, blood loss ≥ 30 mL, mannitol application time ≥ 2 weeks, the use of anticoagulants within 1 week before admission, and surgical treatment were the influencing factors of prognosis of brain contusion and laceration. The details are shown in Table 1.

### 3.3. BPNN Model Analysis of Predictive Variables of Postoperative Prognosis

Based on the BPNN model, the prediction model of poor prognosis of patients with brain contusion and laceration after operation shows that the GCS score < 8 is 65.0 points at admission, the bleeding volume ≥ 30 ml at admission is 80.0 points, the mannitol application ≥ 2 weeks is 87.0 points, the anticoagulants before admission is 100.0 points, and the surgical treatment after admission 24 hours is 71.3 points, as shown in Figure 4.

### 3.4. Comparison of Prediction Model Performance

The receiver operator characteristic (ROC) curve showed that the area under the curve (AUC) of the logistic regression model for predicting the poor prognosis of patients with brain contusion and laceration after the operation was 0.816 (95% *CI* 0.705~0.926). The AUC of the BPNN model is 0.819 (95% *CI* 0.708~0.931). The ROC is shown in Figure 5.

## 4. Discussion

With the development of social modernization and the improvement of economic level, the number of patients with TBI caused by traffic accidents is increasing. The head and neck are some of the most seriously injured organs in traffic accidents [20]. Patients with mild traumatic brain injury can show signs and symptoms of unconsciousness or unconsciousness, forgetfulness, vomiting, or diffuse headache. The disease may develop rapidly in severe cases, leading to irreversible severe disability or death [21]. Brain contusion and laceration are the terms of brain contusion and laceration. Severe contusion and laceration of the brain often complicated with a cerebral hernia are a typical critical illnesses, and patients are often accompanied by obvious neurological impairment. Operation is an important treatment strategy. According to the relevant survey data, the prognosis of patients is generally unsatisfactory, with a high disability rate and mortality rate [22]. The key step to improving the prognosis of patients with brain contusion and laceration is to accurately determine the risk factors that affect the poor prognosis of patients after craniotomy.

The article "Construction and Evaluation of Prognosis Prediction Model for Patients with Brain Contusion and Laceration Based on Machine Learning" was published in 2022. Journal: Comput Math Methods Med.

Brain contusion and laceration are a common primary TBI. Clinically, the diagnosis of brain contusion and laceration is mainly based on the history of TBI, the findings of clinical physical examination, the results of the imaging-assisted examination, and comprehensive analysis combined with the experience of clinicians [23, 24]. CT, MRI, and other imaging examinations provide objective imaging data for clinical diagnosis of cardiovascular and cerebrovascular diseases [25]. However, these imaging findings are also very different at different stages of the disease [26, 27]. To judge the prognosis more accurately, it is necessary to consider the related factors as much as possible.

In this study, the patients with brain contusion and laceration admitted to our hospital in recent years were selected as the research object. The prediction model was built based on logistic regression and BPNN. The clinical data of the two groups of patients were retrospectively analyzed. The details of age, gender, the volume of brain contusion and laceration, blood loss, GCS score of patients admitted to hospital, and treatment methods were sorted out and analyzed, to predict the prognosis of patients after operation. In this study, we concluded that GCS score < 8 on admission, blood loss ≥ 30 ml on admission, mannitol application ≥ 2 weeks, anticoagulants before admission, and surgical treatment were five high-risk factors for poor prognosis after brain contusion and laceration. This study showed that the weight of the model score was 87.0 when mannitol was used for ≥2 weeks. Mannitol is a commonly used drug in clinical practice. Relevant literature reports that using the appropriate amount of mannitol at the right time is helpful to quickly improve cerebral vascular circulation, significantly reduce the degree of brain edema damage, and protect neurological function [28, 29]. Santing et al. [30] demonstrated that TBI is an independent factor of venous vascular embolism. It is a vital link for clinical treatment of TBI to prevent venous vascular embolism by formulating scientific preventive strategies effectively. It is also pointed out that although anticoagulants can prevent venous thrombosis, they may increase the risk of bleeding. In addition, Shehadeh et al. [31] believed that reducing the lesion volume and improving the survival rate of neurons play an essential role in improving the prognosis of brain contusion and laceration. Our research results are consistent with these previous studies.

The article "Construction and Evaluation of Prognosis Prediction Model for Patients with Brain Contusion and Laceration Based on Machine Learning" was published in 2022. Journal: Comput Math Methods Med.

This study verified the prediction model of poor prognosis of patients with brain contusion and laceration. The logistic regression model and the BPNN prediction models predict the poor prognosis of patients with brain contusion and laceration. The areas under the curve are 0.816 (95% *CI* 0.705-0.926) and 0.819 (95% *CI* 0.708-0.931), respectively. This result shows that the established prediction model has good discrimination, but the BPNN model has better predictive efficiency than the logistic regression model.

## 5. Conclusion

This study builds a prediction model based on the risk factors that affect the poor prognosis of patients with brain contusion and laceration, with good discrimination and accuracy. The number of cases included in this study is small, and the promotion of this prediction model still needs to be verified by large-scale and multicenter prospective studies. In future research work, it is also suggested to further screen the independent risk factors of poor prognosis in patients with brain contusion and laceration and continuously optimize the prediction model to better serve the clinical decision-making.

## Figures and Tables

**Figure 1:** Classical BPNN structure diagram.

**Figure 2:** Modeling flow chart of machine learning.

**Figure 3:** Comparison of clinical data of patients with brain contusion and laceration in the training and test sets. There was no statistically significant difference between the two sets (*P* > 0.05).

**Figure 4:** Characteristic factors of poor prognosis in patients with brain contusion and laceration after operation.

**Figure 5:** ROC curve of poor postoperative prognosis in patients with brain contusion and laceration.

**Table 1:** Logistic regression analysis of prognostic factors in patients with brain contusion and laceration.

Factors	SE	*P*	OR	95% CI
Volume of brain contusion	0.631	0.025	2.902	1.182-7.123
GCS scores ≤ 8	2.015	0.023	2.757	1.152-6.600
Amount of bleeding ≥ 30 mL	0.591	<0.001	5.935	2.246-15.683
Mannitol application time ≥ 2 weeks	0.408	0.003	4.164	1.648-10.517
Use of anticoagulants	0.614	0.003	4.017	1.592-10.139
Surgical treatment	0.315	0.002	4.943	1.821-13.417

The article "Construction and Evaluation of Prognosis Prediction Model for Patients with Brain Contusion and Laceration Based on Machine Learning" was published in 2022. Journal: Comput Math Methods Med.

## Data Availability

All data analyzed during this study are available from the corresponding author on reasonable request.
